The article "Impact of Physical Activity and Medication Adherence on the Seizure Frequency and Quality of Life of Epileptic Patients: A Population Study in West Texas" was published in 2022. Journal: Biomed Res Int.

# Impact of Physical Activity and Medication Adherence on the Seizure Frequency and Quality of Life of Epileptic Patients: A Population Study in West Texas

**DOI:** 10.1155/2022/4193664

**Published:** 2022-01-18

**Authors:** YoonJung Lee, Yeseul Ahn, Luca Cucullo

**Affiliations:** ^1^Department of Pharmaceutical Sciences, Jerry H. Hodge School of Pharmacy, Texas Tech University Health Sciences Center, Amarillo, TX 79106, USA; ^2^Department of Foundation Medical Studies, Oakland University William Beaumont School of Medicine, Rochester, MI 48309, USA

## Abstract

Epilepsy is a neurological disease that affects 1-3% of the population. People with epilepsy (PWE) have poor physical and psychological health and a lower quality of life (QOL) than people without epilepsy. Moreover, PWE has more comorbid conditions (obesity, depression) than general populations. Physical activity (PA) has been reported to have various positive physical and psychological effects in PWE. Meanwhile, poor medication adherence is one of the main precipitating factors for seizure triggers. This study assessed the impact of PA and medication adherence on the seizure frequency and QOL for PWE at the Epilepsy Foundation, West Texas (EFWT). Our results indicate that PA is positively associated with the quality of life and negatively associated with the seizure frequency for PWE at EFWT, which suggests that physically active PWE tend to have fewer seizures and better QOL. Medication adherence did not affect the seizure frequency or QOL in our study. Yet, it is still crucial to encourage medication adherence for PWE since nonadherence is a known seizure promoter. Findings from this study highlight the continuous need to utilize available resources and implement programs to promote physical activity and medication adherence for better seizure control and QOL in PWE at EFWT.

## 1. Introduction

Epilepsy is one of the most common neurological diseases globally, affecting 1-3% of the population, 50 million worldwide, and 5.1 million in the U.S. [1–3] Epilepsy is a neurological syndrome defined by having two or more spontaneous, unprovoked seizures separated by at least 24 hours [4]. An epileptic seizure is a transient occurrence of signs and symptoms due to abnormal excessive or synchronous neuronal activity in the brain [4, 5]. Focal and generalized seizures are the two main types of seizures, where generalized tonic-clonic seizures involve a loss of consciousness with generalized body stiffening and jerking [6]. People with epilepsy (PWE) develop cognitive dysfunction over time as the disease progresses [7, 8]. Furthermore, PWE experience several adverse drug events related to the use of antiepileptic drugs (AEDs), such as weight gain, osteoporosis, fatigue, drowsiness, and other side effects [9–12].

Besides the negative impact of epilepsy on physical health, epilepsy-related stigma negatively impacts an individual's life, including economic and employment status, psychological well-being, social interactions, self-esteem, and overall health [13]. Furthermore, several studies reported epilepsy-related stigma to influence medication adherence negatively [14, 15]. Medication adherence rate for PWE ranges between 30% and 60%, with an indirect correlation between the degree of disease-related stigma and medication adherence [16–18]. PWE with higher levels of disease-related stigma have lower medication adherence and poor compliance to medication, which may lead to precipitated seizures [15, 19].

PWE, with lifestyle restrictions, have more comorbid conditions than general populations. 27% to 84% of PWE have at least one comorbid medical condition, and nearly every PWE will experience a comorbid medical condition at some point during the treatment [20, 21]. Comorbid conditions that are significantly higher in PWE than general populations include medical diseases (e.g., musculoskeletal disorders, chronic pain disorders, migraine, arthritis, obesity, fractures), psychiatric diseases (e.g., depression and anxiety), and cognitive diseases (e.g., ADHD and learning disability) [21].

When all these factors (e.g., seizures, adverse drug events from AEDs, stigma, other comorbidities, and lifestyle restrictions) are summed up together, they negatively affect the overall quality of life (QOL) of PWE. As a result, PWE have a lower QOL than people without epilepsy [22, 23]. PWE especially have lower scores in physical and psychosocial areas. This observation is potentially due to epilepsy-associated lifestyle restriction and epilepsy-related stigma that leads to lower self-esteem and higher rates of anxiety and depression [24, 25].

Physical activity (PA) is defined as any bodily movement produced by skeletal muscles in daily life that results in energy expenditure and can be categorized into occupational, sports, conditioning, household, or other activities [26]. PA has various positive physical and psychological effects in PWE. In terms of PA's positive physical effect in PWE, one potential explanation is physical activity promoting general health, well-being, and improving cardiovascular function, thereby aiding to manage physical comorbidities (obesity) commonly observed in PWE [27]. Additionally, PA can exert positive psychological effects by improving mood and reducing stress, one of the most frequently self-reported precipitants of seizure, in PWE [27]. The beneficial effects of PA include comorbidity management, reduction in adverse drug events by antiepileptic drugs, overall improvements in health, QOL, and behavioral outcomes [22, 27–30]. For example, a study conducted by Volpato et al. reported better QOL and lower seizure frequency when PWE had higher physical activity and aerobic capacity [22]. Another study by Hafele et al. reported a positive association between PA and QOL and negative associations between PA and depression, anxiety, and adverse effects of medication in PWE [30]. Limited studies also evaluated the effects of PA in seizure frequency. These studies had mixed results, with a significant decrease in seizure frequency reported in three studies, no change in seizure frequency in the remaining studies [22, 29, 31–33]. None of the studies reported increased seizure frequency during the exercise programs. The exact mechanism of how physical activity helps to reduce seizures is unknown. Still, a few potential mechanisms of physical activity reducing seizures include (1) PA to reduce neuroinflammation, which is a known trigger for epilepsy, and (2) improved mitochondrial function to generate more energy sources for neurons, which helps for stabilization of neuronal activity [34–36].

Furthermore, all of these studies reported positive outcomes of PA. These positive outcomes include increased physical capacity and improvement in QOL, general health, psychological state, and emotional status [22, 29, 31–33]. Up to date, there is only one study that has evaluated the association between physical fitness and the risk of epilepsy at a later life. A prospective Swedish study conducted on male participants (*n* = 1,173,079) analyzed the association between cardiovascular fitness at age 18 years and the future risk of epilepsy [37]. In this study, low cardiovascular fitness early in life was associated with an increased risk of epilepsy later in adulthood, with people in low cardiovascular fitness at almost twice an increased risk of having epilepsy compared to people in high cardiovascular fitness [37]. Yet, further extensive and additional studies are required to confirm this observation.

Discouraging PA in PWE has been the norm in the past. In 1968, the American Medical Association (AMA) recommended restricting PWE from engaging in physical activity due to fear of fall injury or exercise-induced seizures [28]. Even after AMA officially removed this restriction, PWE tend to be less active than the general population [38, 39]. Furthermore, PWE have both common barriers (e.g., lack of time and motivation) to engage in PA observed in general people and additional barriers of engaging in PA, such as fear of seizure occurrence, fear of seizure-related injuries, and incorrect advice from medical professionals [40]. As a result, obesity remains one of the most common comorbidities reported in PWE.

With a recent shift in medical recommendations to encourage sports participation in PWE, International League Against Epilepsy (ILAE) Task Force offered general guidance for the involvement of PWE in sports activities by dividing sports activities into three categories [41]. These categories are based on the potential risk of injury or death, with group 1 sports with no significant additional risk and group 3 sports with major risk [41]. Furthermore, the development of the seizure monitoring device can encourage physical activity in PWE. Embrace is the first seizure detection device that received clearance from the FDA in 2018. This device monitors the generalized tonic-clonic seizures and sends an alert to summon caregivers' help. Embrace detects seizure by a combination of two systems: (1) Accelerometry (ACM) monitoring system that detects wrist acceleration and vibration during the seizure attack and (2) electrodermal activity (EDA) monitoring system that quantifies physiological changes related to the sympathetic nervous system activity. The device alerts the caregivers only when there is a combination of the seizure involving convulsive movements and a spike in autonomic stress with ≥20 seconds duration [42]. Yet, up to date, no data is available that has assessed PWE's awareness of this device.

The beneficial effects of PA in PWE have been well reported in studies by Volpato et al. and Hafele et al. [22, 30] In this study, we wanted to assess the impact of PA and medication adherence on seizure frequency and QOL. The primary outcome of the program evaluation project was to evaluate the effect of PA and medication adherence on seizure frequency and QOL for PWE at the Epilepsy Foundation, West Texas. Additionally, we have compared male patients and female patients to assess any gender differences for our findings. The secondary outcome of our project was to obtain the demographic information of PWE, to assess PWE's perception regarding physical activity, potential barriers of physical activity, PWE's awareness on the seizure detection device, seizure types, and seizure frequencies, and to assess the areas of care that potentially require an improvement for PWE at the Epilepsy Foundation, West Texas (EFWT).

## 2. Methods

### 2.1. Setting and Study Population

Epilepsy Foundation, West Texas, is one of the regional offices of the Epilepsy Foundation Texas (EFTX) that provides programs and services for PWE living in the West Texas area, including Amarillo and Lubbock. The programs and services offered include medical clinics staffed by a neurologist, nurse, social worker, prescription assistance, information and referral services, and education programs. Currently, about 150 registered patients receive care from this foundation. Participation in this study was solely voluntary and did not affect the current care treatment of the patient in either case. The EFWT staff responsible for checking in patients for on-site care conducted a survey only for patients who voluntarily agreed with verbal consent. Also, patients had full authority to answer or not answer any of the survey questions. None of the survey questions contained identifiable patient information per HIPAA guidelines.

Additionally, all patient data were deidentified before the data analysis process to ensure confidentiality. Since this project was a program evaluation project without direct patient intervention, the TTUHSC Quality Improvement Review Board determined this project as a program evaluation project. Thus, this project did not require a further institutional review.

### 2.2. Assessment of Demographic Information, Physical Activity, Quality of Life, and Medication Adherence

#### 2.2.1. Demographic Information

We requested a patient to fill out the physical survey form voluntarily for data collection. Inclusion criteria were adult patients (≥18 years old) currently receiving medical treatment at Epilepsy Foundation, West Texas. Exclusion criteria were pediatric patients (<18 years old), an intellectual disability, or other health conditions limiting their capacity to complete the self-administered survey. The survey consisted of 79 total questions that assessed four different areas: demographic information, physical activity, quality of life, and medication adherence. A survey was available in both English and Spanish. For demographic data, there were 20 questions to obtain basic information, health-related information, perception of physical activity and seizure detection device, characteristics of seizures, current antiepileptic drugs (AEDs), and other prescription or over-the-counter drugs, and a patient self-reported seizure frequency. For seizure frequency, we used the median seizure frequency [43]. We obtained the survey instruments from the Social and Behavioral Instruments (SABI) database [44], which provides the validated measurement instruments to the researcher to assess physical activity, quality of life, and medication adherence. International Physical Activity Questionnaire (IPAQ)-long version, World Health Organization Quality of Life-BREF (WHOQOL-BREF), and Simplified Medication Adherence Questionnaire (SMAQ) were the three survey instruments utilized because of their validity and reliability established from multiple studies with extensive use in various settings [45–47].

#### 2.2.2. Quantification and Categorization of Physical Activity

We used an IPAQ-long version to measure physical activity in people with epilepsy [45]. IPAQ assesses physical activity in the set of domains, including leisure-time physical activity, domestic and gardening (yard) activities, work-related physical activity, and transport-related physical activity. Then, after calculating Metabolic Equivalent Task minutes per week (MET-minutes/week), physical activity variables were categorized as follows: (1) Low—no activity or some activity reported, but not enough to meet moderate or high categories. (2) Moderate—either one of the following three categories: (a) 3 or more days of vigorous-intensity activity of at least 20 minutes per day OR (b) 5 or more days of moderate-intensity activity and/or walking of at least 30 minutes per day OR (c) 5 or more days of any combination of walking, moderate-intensity, or vigorous-intensity activities achieving a minimum of at least 600 MET-min/week. (3) High—any one of the following two criteria: (a) vigorous-intensity activity on at least three days and accumulating at least 1500 MET-minutes/week OR (b) 7 or more days of any combination of walking, moderate-, or vigorous- intensity activities accumulating at least 3000 MET-minutes/week. Patients who reported exercising ≥16 hours per day were excluded under the assumption that an individual requires 8 hours per day for sleeping.

#### 2.2.3. Assessment of Quality of Life

World Health Organization Quality of Life-BREF (WHOQOL-BREF), a short version of the WHOQOL-100, was used to assess QOL in PWE. The choice of survey tool was made to compare QOL between PWE and people without epilepsy. Unlike the Quality of Life in Epilepsy Inventory (QOLIE), which can only be administered in PWE, WHOQOL-BREF is a nondisease-specific tool with broader application.

The questionnaire consists of a total of 26 questions, 24 questions to assess four domains (physical health, psychological health, social relationships, environment), and two questions to evaluate an individual's overall perception of his quality of life (overall QOL) and an individual's overall perception of his health (general health) [46]. The answers ranged on a scale of 1 to 5, with higher scores reporting better QOL, except for three negatively phrased questions with higher scores indicating lower QOL [46]. The raw score of each domain was calculated and then transformed into a 0-100 scale for an individual patient using an equation and table from the WHOQOL-BREF manual. After obtaining the study participants' average, we compared these numbers to the WHOQOL US average QOL scores for healthy subjects and chronically ill patients reported in the literature [48].

#### 2.2.4. Assessment of Medication Adherence

We utilized the Simplified Medication Adherence Questionnaire (SMAQ) that consists of 6 items designed to assess medication adherence [47]. In this survey, a positive response to any of the qualitative questions indicates a nonadherence to the medication. These qualitative questions include (1) ≥2 doses missed over the past week and (2) ≥ two days of not taking any medication during the past three months [47].

### 2.3. Statistical Analysis

A descriptive analysis of the collected data was carried out using Excel 2013 to organize and evaluate the demographic information, MET-minutes/week, physical activity categories (low, moderate, and high), quality of life domain scores, and medication adherence rate. Statistical analysis was carried out by GraphPad Prism 8 (GraphPad Software Inc., San Diego, California, USA). Spearman's correlation test was used to evaluate the correlation between physical activity based on MET-minutes/week and the seizure frequency. ANOVA test followed by Dunn's multiple comparisons test was used to compare the seizure frequency between three groups with different physical intensity categories (low, moderate, and high). Pearson's correlation test was used to evaluate the correlation between physical activity and the six parameters of quality of life. ANOVA test followed by Tukey's test was used to compare the quality of life between three groups (people with epilepsy, chronically ill patients, and healthy individuals) and compare the quality of life between three groups with different physical intensity categories. A Student's unpaired *t*-test was used to compare the seizure frequency between the medication adherent and nonadherent groups.

## 3. Results

A Total of 24 Surveys Were Collected in the Study: The Findings of our Study Are Summarized in Figures 1–5

### 3.1. Physical Activity and Seizure Frequency

Five PWE were in the low physical activity category, eight PWE were in the moderate physical activity category, and six PWE were in the high physical activity category. Overall, there was a moderate negative correlation between physical activity (MET-minutes/week) and seizure frequency, indicating physical activity to be associated with lower seizure frequency (*r* = −0.5266, Spearman's correlation test, Figure 1(a)). PWE in the high physical category had substantially lower seizure frequency than the other two groups (low and moderate physical categories) without statistical significance (one-way ANOVA test and Dunn's multiple comparison test) (Figure 1(b)).

### 3.2. Physical Activity (PA) and Quality of Life (QOL)

Overall, there was no correlation between PA and domain 3 (social), with weak correlations between PA and domain 1 (physical), PA and domain 2 (psychosocial), and PA and domain 4 (environment) without statistical significance (*r* = 0.3023, *p* = 0.2228, Figure 2(a); *r* = 0.3194, *p* = 0.1963, Figure 2(c), *r* = 0.3508, *p* = 0.1535, Figure 2(d), *r* = −0.0919, *p* = 0.7257, Figure 2(e), *r* = 0.2839, *p* = 0.2537, Figure 2(f)). For overall health, there was a moderate positive correlation with statistical significance between physical activity (MET-minutes/week) and seizure frequency (*r* = 0.5388, ^∗^*p* = 0.0210, Pearson's correlation test, Figure 2(b)).

### 3.3. Quality of Life

QoL scores for PWE were similar to the general QOL scores of the chronically ill patients in the U.S. One-way ANOVA test followed by Tukey's comparison has demonstrated PWE patients to have significantly lower scores than healthy patients in the U.S. for all parameters of QOL except the overall QOL (Figure 3(a)).

Among PWE, when we compared QOL scores between three groups with different exercise intensities, PWE in the high physical activity category had substantially higher QOL scores than the other two groups. One-way ANOVA test followed by Tukey's comparison has demonstrated PWE with high physical activity having significantly higher scores than the other two groups in two domains, psychosocial health (^∗^*p* = 0.0416) and environment (^∗^*p* = 0.0349) (Figure 3(b)).

### 3.4. Medication Adherence

Fifty-two percent of patients were adherent to medication, and forty-eight percent were nonadherent (Figure 4(a)). There was no difference in seizure frequency between the medication adherent and nonadherent groups (Student's unpaired *t*-test, Figure 4(b)) There was no difference in medication adherence for PWE with different physical activity intensities (Student's unpaired *t*-test, Figure 4(c)). There was no difference in QOL in the medication adherent group versus the nonadherent group (Student's unpaired *t*-test, Figure 4(d)).

### 3.5. Male vs. Female

There was no difference in seizure frequency between the two groups (Figure 5(a)). There was no difference in physical activity (MET per week) between the two groups (Figure 5(b)). There was no difference in the number of patients with different exercise intensities (low, moderate, and high) per group (Figure 5(c)). There was no difference in medication adherence between the two groups (Figure 5(d)). There was no difference in QOLs for all parameters between the two groups (Figure 5(e)).

### 3.6. Characteristics of People with Epilepsy (PWE)

The characteristics of the participants are summarized in Tables 1(a)–1(d).

Basic information: the demographic information (age, gender, marital status, ethnicity, health insurance status, education, occupation, and income level) and obesity status are listed in Table 1(a). The collected information suggested patients' age in a wide range (19-70 years old), more males than females, nearly half of patients having obesity and unmarried, and the majority of patients being either White or Hispanic. In terms of socioeconomic factors, most patients were underinsured, had lower education levels, were unemployed, and had low to no income.

Health-related information: most common comorbidities were arthritis, hypertension, asthma, and migraine/headache. A small number of respondents had mental illnesses (bipolar disorder, anxiety, and depression). More than one-third of the PWE were smokers. Since some patients had ≥2 conditions, the final percentage was not equal to 100% (Table 1(b)).

Perception of physical activity and seizure detection device: almost all PWE acknowledged the importance of exercise (>90%). Half of the patients responded to exercise regularly. Walking and yard work were the most preferred exercise. Also, the patients reported several potential barriers to exercise. Most patients (92%) were unaware of seizure detection devices (embrace). Major barriers to purchasing seizure detection devices were the cost and uncertainty (Table 1(c)).

Types of seizures, current antiepileptic drugs (AEDs), and self-reported seizure frequency: the patients had various first onset of the seizure, with more than half of the patients experiencing seizure before age 18. Some patients reported having ≥2 types of seizures, which made the final percentage not equal to 100%. Complex focal seizures and tonic-clonic seizures were the most common type of seizures. About one-third of patients did not know the type of seizure they had. Most patients had <50 seizures per year, with one patient having 180 seizures per year. Few patients could not report their seizure frequency. Carbamazepine, valproic acid, and levetiracetam were the top three most prescribed anticonvulsants. Most patients were on one to two anticonvulsants (>70%). A few patients could not recall their current anticonvulsants (Table 1(d)).

## 4. Discussion

For our project, we designed our study to evaluate the effect of PA on seizure frequency, QOL, and medication adherence simultaneously for PWE at the EFWT. Additionally, we have obtained the demographic information, PWE's perception regarding physical activity, potential barriers to physical activity, and PWE's awareness of the seizure detection device. We have successfully achieved our primary and secondary outcome measurement through data collection of self-reported surveys and data analysis. Additionally, this project helped us assess the areas of care that potentially require improvement for PWE at the EFWT.

Overall, there was a statistically significant moderate negative correlation between physical activity (MET-minutes/week) and seizure frequency. This observation indicates that PWE who are physically active tend to have fewer seizures. Also, PWE in the high physical activity category had substantially lower seizure frequency than the other two groups with different physical intensities (low and moderate). Though there was no statistical significance, this could be due to a small sample size per group. Therefore, our overall results indicate an association between physical activity and seizure frequency in PWE.

The existing literature reported that physical activity was positively associated with QOL in PWE. For example, Hafele et al. reported a positive correlation between the amount of physical activity and QOL score in PWE [30]. Additionally, Volpato et al. reported physically active PWE having higher overall QOL than physically inactive PWE [22]. Our findings on physical activity and overall health matched this existing literature. As demonstrated in Figure 2(b), physical activity and overall health were the sole parameter of QOL with a statistically significant moderate positive correlation. As reported in the existing literature, our result indicates highly active PWE tend to have a better perception of their overall health than PWE with lower physical activity.

When Bonomi et al. conducted a study to validate the U.S. version of the WHOQOL, chronically ill patients with ≥1 chronic condition for ≥1 year and received medical care for the condition had lower QOL than healthy adults [48]. In this lieu, for our study, it is not surprising to discover PWE with ≥1 chronic condition (e.g., epilepsy and other comorbidities) to have a similar QOL score as the chronically ill patients in the U.S. (Figure 3). Additionally, as reported in the existing literature, PWE in our study had significantly lower QOL scores than healthy individuals in the U.S. This observation is due to having comorbidity negatively affecting QOL. Yet, for QOL scores in PWE with different physical activity intensities (low, moderate, and high), highly active PWE had substantially higher QOL scores than the other groups. Also, this group had a statistically significant higher score in two domains (psychosocial health, environment) than the other two groups. Considering physical activity has a positive effect on psychological health (e.g., lowering anxiety and depression in PWE), this finding also matches up with the results from the existing literature and confirms the positive effect of PA on QOL in PWE [22, 30].

Overall, 52% of PWE were adherent to medication. This percentage falls within the usual medication adherence range for PWE [16–18]. Despite two patients with the most and the second most seizure frequencies in the nonadherent group, no difference in seizure frequency was observed between the medication adherent and medication nonadherent groups. This result contrasts the existing literature that has reported nonadherence to the anticonvulsants as one of the main precipitating factors for seizure triggers [49–51]. A low number of data collection for this survey is a potential explanation for this observation.

No difference in the QOL scores was observed between medication adherent and nonadherent groups. This result contrasts the several studies that have reported a positive association between medication adherence to anticonvulsants and QOL [52, 53]. Having one or more comorbidities for most PWE in our study could have an additional negative effect on the QOL for PWE at EFWT, which might not be attenuated by medication adherence alone. For example, a study that has reported a positive association between medication adherence and QOL only included PWE without any other comorbidities [53].

There was no difference in seizure frequency, physical activity, intensity, medication adherence, and QOLs between male and female subjects.

Demographic information, one of the secondary outcome measurements, helped us identify common comorbidities in PWE at EFWT. Obesity is reported by half of the survey respondents (47%) and was one of the most common comorbidities, followed by arthritis and hypertension for PWE at EFWT. This finding matches the existing literature, which has reported higher comorbidities (obesity, arthritis, and hypertension) in PWE than the general population [54–58]. The potential causes of higher obesity in PWE than the general population include physical inactivity and adverse events from AED. Besides physical inactivity well known to contribute to obesity, certain anticonvulsants (e.g., gabapentin, pregabalin, valproic acid, and vigabatrin) stimulate appetite and induce sedation and lethargy, which lead to decreased physical activity and weight gain [59]. Additionally, since obesity is the known major risk factor for both hypertension and arthritis, including osteoarthritis and rheumatoid arthritis, this was an expected finding that 71% of the survey respondents with arthritis and 75% of the survey respondents with hypertension were either overweight or being obese [60–62]. Regarding physical activity, most PWE valued the importance of exercising (>90%), with half of PWE at EFWT attempting to exercise regularly. Exercise preference was primarily geared toward physical activities with a low risk of fall injuries such as walking and yard work. Physical disability or other disease conditions, fear of fall injury, the uncertainty of suitable exercise, and hard-to-find time for exercise were the most commonly reported potential barriers to exercise and were in line with reported in the literature [38, 40].

Only a few people were aware of the seizure detection device (Embrace). Furthermore, even people aware of the seizure detection device were uncertain how this device works and reluctant to purchase the device due to its high cost that could be due to the PWE at EFWT having low socioeconomic status with zero to low income. As a result, the price of a device ($249) and a monthly subscription fee that ranges between $9.90 and $44.90 may not be affordable for PWE unless there is a form of financial assistance such as Medicare.

This project helped us identify the areas of care that potentially require improved PWE at the EFWT. Though most people acknowledged the importance of physical activity, specific potential barriers such as fear of fall injury and uncertainty for suitable exercise exist in PWE and make them less physically active. An exercise promoting programs such as Get FIT Texas has the potential to overcome these barriers under supervision by trained healthcare professionals [63]. From 2012 to 2017, this program provided fitness and healthy lifestyle coaching to PWE from the Epilepsy Foundation. PWE enrolled in this program had very favorable outcomes, such as 80% of the participants with improvement in BMI score, and 90% of participants scored higher on their quality of life tests after completion of the program. Therefore, reinstating the exercise program for PWE can improve both physical health and overall QOL in PWE.

Medication adherence and medication education are other areas of care that require improvement for PWE at the EFWT. In our study, almost half of the study participants were nonadherent to the medications. Furthermore, people had virtually little to no knowledge of other prescription medications, over-the-counter (OTC) drugs, or herbal supplements. To improve medication adherence, some resources to encourage medication adherence, such as My Seizure Diary and Texting 4 Control, the app, and a text message system designed to enhance medication adherence, can be utilized. Medication education or reconciliation programs can better the therapeutic management and reduce the risk of drug interactions [49, 64, 65].

Overall, PWE at EFWT had lower QOL than people without epilepsy. This finding is not surprising, considering epilepsy is reported to impact PWE's QOL negatively [22, 23]. Yet, it is good to observe QOLs be positively associated with a level of physical activity for PWE. Though there was no significant difference in QOLs for medication adherent PWE versus medication nonadherent PWE in our study, poor compliance with an anticonvulsant is the leading cause of the precipitated seizures and has a negative influence on QOLs of PWE. Therefore, it is essential to evaluate the QOLs regularly for PWE at EFWT and monitor other factors such as medication adherence and physical activity, the two factors known to influence QOLs of PWE.

### 4.1. Limitations

For this study, the data was collected from the EFWT. Therefore, the demographic information may differ for PWE reside in other regions. A low response rate, which was 12% (24 responses out of 150 patients), is a limitation of this study. Only limited patients were willing to answer the survey. Providing a form of small compensation may increase the response rate for future studies. It would have been surplus if seizure frequency was obtained using more accurate methods (e.g., electroencephalogram (EEG) and video-based telemetry). Yet, considering our study being an assessment study, it may be less crucial to obtain seizure frequency using objective method. Thus, subjective method such as a self-reported seizure frequency is still acceptable for our study. Still, our study is significant in a way that has evaluated the effect of PA and medication adherence on the QOL and seizure frequency of the PWE.

## 5. Conclusion

In conclusion, physical activity is positively associated with the quality of life and negatively associated with the seizure frequency for PWE at EFWT. However, unlike existing literature, there was no association between medication adherence and seizure frequency or QOL. The findings from this assessment study will be beneficial for EFWT to think of implementing certain programs (e.g., Get FIT Texas) to promote the well-being of the patients.

## Figures and Tables

**Figure 1:** (a) Physical activity (MET) versus seizure frequency per year (*r* = −0.5266, ^∗^*p* = 0.0380, moderate negative correlation, Spearman's correlation test). The result indicates that physically active people tend to have fewer seizures. (b) Comparison of seizure frequency in PWE with three different exercise intensities (one-way ANOVA test, NS for all three groups with *p* > 0.999 for low vs. moderate, *p* = 0.1406 for low vs. high, *p* = 0.2420 for moderate vs. high).

**Figure 2:** (a–f) Physical activity (MET) versus QOL score of six parameters. Pearson's correlation test (*r* = 0.3023, *p* = 0.2228 (a); *r* = 0.5388, ^∗^*p* = 0.0210 (b); *r* = 0.3194, *p* = 0.1963 (c), *r* = 0.3508, *p* = 0.1535 (d), *r* = −0.0919, *p* = 0.7257 (e), *r* = 0.2839, *p* = 0.2537 (f).

**Figure 3:** (a) Assessment and comparison of QOL in three groups (PWE, chronically ill, healthy individuals). Data for chronically ill patients and healthy individuals are obtained from literature to compare with PWE (^∗^*p* < 0.05, ^∗∗^*p* < 0.01, ^∗∗∗^*p* < 0.001, ^∗∗∗∗^*p* < 0.0001, one-way ANOVA test). (b) Assessment and comparison of QOL in three groups with different exercise intensities (^∗^*p* < 0.05, ^∗∗^*p* < 0.01, ^∗∗∗^*p* < 0.001, ^∗∗∗∗^*p* < 0.0001, one-way ANOVA test).

**Figure 4:** (a) Assessment for the percentage of adherent versus nonadherent to medication in PWE. (b) Assessment of medication adherence versus seizure frequency. Student's unpaired *t*-test (*p* = 0.6051). (c) Assessment of physical adherence versus medication adherence. Fisher's exact test (*p* > 0.9999 for all groups). (d) Assessment and comparison of QOL in two groups (adherent versus nonadherent). Student's unpaired *t*-test (*p* = 0.4439 (overall QOL), *p* = 0.5053 (overall health), *p* = 0.5796 (physical health), *p* = 0.5821 (psychosocial health), *p* = 0.5681 (social relationship), *p* = 0.6913 (environment)).

**Figure 5:** (a) Comparison of seizure frequency in two groups (male versus female). Mann-Whitney test (*p* = 0.4711). (b) Comparison of MET-per week in two groups (male versus female). Student's unpaired *t*-test. (*p* = 0.7456). (c) Number of patients with different exercise intensities (low, moderate, and high) per group. Fisher's exact test (*p* > 0.9999 for moderate vs. high, *p* = 0.1818 for low vs. high, *p* = 0.2308 for low vs. moderate). (d) Comparison of medication adherence between two groups (male versus female). Fisher's exact test (*p* = 0.3964). (e) Assessment and comparison of QOL in two groups (male versus female). Student's unpaired *t*-test (*p* = 0.3069 (overall QOL), *p* = 0.7854 (overall health), *p* = 0.2756 (physical health), *p* = 0.3776 (psychosocial health), *p* = 0.3872 (social relationship), *p* = 0.7589 (environment)).

**Table 1a:** (a) General demographic information: basic information

	People with epilepsy (total *n* = 17‐24^∗^, %)
Mean age ± SD (range)	39 ± 14 (19–70)
Gender	
Male	10/24 (42%)
Female	14/24 (58%)
Body mass index (BMI)	
Underweight (≤18.5)	1/17 (6%)
Normal weight (18.5–24.9)	6/17 (35%)
Overweight (25–29.9)	2/17 (12%)
Obese (≥30)	8/17 (47%)
Obese class I (30.0-34.9)	4/17 (24%)
Obese class 2 (35-39.9)	2/17 (12%)
Obese class 3 (≥40)	2/17 (12%)
Marital status	
Single	12/24 (50%)
Married	5/24 (20.8%)
Divorced	4/24 (16.7%)
Engaged or in a relationship	3/24 (12.5%)
Ethnicity	
White or Caucasian	14/24 (58.3%)
Hispanic or Latino	7/24 (29.2%)
Asian	1/24 (4.2%)
Black or African American	1/24 (4.2%)
Other (mixed, White, and Latino)	1/24 (4.2%)
Health insurance	
Yes (e.g., Medicaid, JOWYATT)	14/24 (58.3%)
No	10/24 (41.7%)
Education	
High school diploma or GED	17/24 (70.8%)
Some college credits	3/24 (12.5%)
Associate degree from college	1/24 (4.2%)
Bachelor's degree from college	3/24 (12.5%)
Occupation	
Employed	6/24 (25%)
Unemployed (e.g., homebound)	17/24 (70.8%)
Student	1/24 (4.2%)
Income level	
$0-$5000	15/24 (62.5%)
$5000-$10,000	1/24 (4.2%)
$10,000-$20,000	4/24 (16.7%)
$20,000-$30,000	2/24 (8.3%)
$30,000-$40,000	2/24 (8.3%)

^∗^For some questions, not all of them responded to the questions.

**Table 1b:** (b) General demographic information: health-related information

	People with epilepsy (total *n* = 18‐24^∗^, %)
Other health conditions besides epilepsy^∗∗^	
Arthritis	7/18 (38.9%)
Hypertension	6/18 (33.3%)
Asthma	4/18 (22.2%)
Migraine/headache	4/18 (22.2%)
None	3/18 (16.7%)
Liver problems (e.g., cirrhosis, fatty liver)	2/18 (11.1%)
Acid reflux/GERD	2/18 (11.1%)
Type 2 diabetes	2/18 (11.1%)
Heart failure	2/18 (11.1%)
Bipolar disorder	2/18 (11.1%)
Anxiety sensitivity	1/18 (5.6%)
Depression	1/18 (5.6%)
Sleep apnea	1/18 (5.6%)
IGA neuropathy	1/18 (5.6%)
Chronic bronchitis/COPD	1/18 (5.6%)
Hyperthyroidism	1/18 (5.6%)
Smoking	
Yes	9/24 (37.5%)
≤1/2 pack per day	6/24 (25%)
≥1/2 to 1 pack per day	2/24 (8.3%)
Do not know	1/24 (4.2%)
No	15/24 (62.5%)

^∗^For some questions, not all of them responded to questions. ^∗∗^Some patients had ≥2 health conditions.

**Table 1c:** (c) General demographic information: perception of physical activity and seizure detection device

	People with epilepsy (total *n* = 14‐24^∗^, %)
Importance of exercise/physical activity	
Extremely important	1/24 (4.2%)
Very important	6/24 (25%)
Somewhat important	15/24 (62.5%)
Not so important	1/24 (4.2%)
Not at all important	1/24 (4.2%)
Exercise regularly	
Yes	12/24 (50%)
No	12/24 (50%)
Types of exercise	
Walking	8/14 (57.1%)
Running	1/14 (7.1%)
Yardwork	2/14 (14.3%)
Standard exercise	1/14 (7.1%)
No exercise/NA	2/14 (14.3%)
Potential barriers to prevent physical activity^∗∗^	
Fear of fall injury	5/21 (24%)
Uncertainty for suitable exercise	4/21 (19%)
Hard to find time for exercise	3/21 (14%)
Physical disability or other disease conditions	6/21 (29%)
Others (e.g., bad hips, tired/do not feel well, always must have someone with me, joint pain)	5/21 (24%)
Aware of the seizure detection device on the market	
Yes, but do not know the name	1/24 (4.2%)
Yes (e.g., SeizureLink)	1/24 (4.2%)
No	22/24 (91.7%)
Purchased seizure detection device/reasons for not purchasing a device	
Yes	0/2 (0%)
No (e.g., cost, uncertain how it really works)	2/2 (100%)

^∗^For some questions, not all of them responded to questions. ^∗∗^Some patients had ≥2 responses.

**Table 1d:** (d) General demographic information: characteristics of seizures, types, and the total number of anticonvulsants used

	People with epilepsy (total *n* = 21‐24^∗^, %)
Onset of seizure for the first time	
Pediatric and adolescent (age 0-18)	13/24 (54.2%)
Adult (≥18)	9/24 (37.5%)
Unknown/not sure	2/24 (8.3%)
Types of seizures^∗∗^	
Complex focal seizures (loss of consciousness)	10/21 (47.6%)
	5/21 (23.8%)
Simple focal seizures (seizure without loss of consciousness)	7/21 (33.3%)
	10/21 (47.6%)
Generalized seizures (absence seizures)	3/21 (14.3%)
Generalized seizures (tonic-clonic seizures)	1/21 (4.8%)
Generalized seizures: atonic seizures (also known as drop attacks)	6/21 (28.6%)
Unknown/idiopathic	
Other (e.g., nocturnal seizure, do not know)	
Seizure frequencies	
0-10 per year	6/24 (25%)
11-24 per year	6/24 (25%)
25-48 per year	8/24 (33.3%)
60-120 per year	1/24 (4.2%)
180 per year	1/24 (4.2%)
Uncertain/unknown	2/24 (8.3%)
Types of anticonvulsants used^∗∗^	People with epilepsy (total *n* = 21^∗^, %)
Brivaracetam	1/21 (4.8%)
Carbamazepine	8/21 (38.1%)
Clonazepam	2/21 (9.5%)
Eslicarbazepine	2/21 (9.5%)
Lacosamide	1/21 (4.8%)
Levetiracetam	3/21 (14.3%)
Perampanel	1/21 (4.8%)
Phenobarbital	1/21 (4.8%)
Phenytoin	3/21 (14.3%)
Pregabalin	1/21 (4.8%)
Topiramate	1/21 (4.8%)
Valproic acid	4/21 (19.0%)
Zonisamide	1/21 (4.8%)
Total number of anticonvulsants used per patient^∗∗^	
One anticonvulsant	9/21 (42.9%)
Two anticonvulsants	6/21 (28.6%)
Three anticonvulsants	1/21 (4.8%)
Four anticonvulsants	2/21 (9.5%)
Unknown	3/21 (14.3%)

^∗^For some questions, not all of them responded to questions. ^∗∗^Some patients had ≥2 responses.

## Data Availability

The datasets generated and/or analyzed during the current study are available from the corresponding author on reasonable request.
